# Experimental Study on Mechanical Properties of Rebar in Steel Half-Grouted Sleeve Connections with Construction Defects

**DOI:** 10.1155/2022/9379135

**Published:** 2022-08-22

**Authors:** Dong Chen, Zhiyong Zhang, Xiaozhen Liu, Qiong Wang, Baojun Zhao, Gang Ren, Changjun Wang

**Affiliations:** ^1^BIM Engineering Center of Anhui Province, Anhui Jianzhu University, Hefei 230601, China; ^2^Anhui Jianzhu University, Hefei 230601, China; ^3^China State Construction HaiLong Technology Company Limited, Shenzhen, Guangdong 518000, China; ^4^Beijing Building Research Institute Corporation Limited of CSCEC, Beijing 100076, China

## Abstract

A prefabricated concrete structure is a building structure designed for sustainability and low comprehensive carbon emission. The grouted sleeve splice is a major connection method for prefabricated concrete structures. However, construction defects occur easily in the grouted sleeve splice connection at construction sites because of complex construction environments and the high connection accuracy. To determine the influence of rebar in steel half-grouted sleeve connections with construction defects, investigations were conducted using four different test groups (rebar offset, rebar bended, insufficient fluidity of grout, and control group). The load—displacement curve and load—stress curve were analyzed on 24 different specimens through uniaxial tension experiments. The experimental results showed that rebar fracture was the failure of specimens. The load—displacement curves consisted of elastic, yield, strength, and tight stages. The curves were similar to rebar under uniaxial tension, except for the rebar bended group. The axial stress and circumferential stress on the sleeve surface consistently followed a linear response before the specimen yield, whereas the axial stress and circumferential stress showed a rebound response after the specimen yielded. Different finite element models were established based on the different defects. Compared with the experimental results, the finite element analysis results coincided with those of the experimental results, and the errors were within 8% to evaluate the performance of steel half-grouted sleeve connections in construction.

## 1. Introduction

Prefabricated concrete structures are increasingly replacing traditional concrete structures because the former possess considerable advantages, such as a high industrialization level, low construction cost, low labor intensity, and low energy consumption. Currently, the performance of node connection is the main factor that influences the safety of prefabricated concrete structures. Grouted sleeve effectively solves the technical problems of node connection in prefabricated concrete structural members [1–3]. Recently, grouted sleeve connections have been widely used because of their high construction efficiency, absence of welding at construction sites, and easy quality control [4]. The types of grouted sleeve include whole-grouted sleeve and half-grouted sleeve. The half-grouted sleeve is mechanically connected by the connected rebar of the upper component at one end, while the embedded rebar of the lower component at the other end is inserted into the sleeve cavity, which is connected by injecting high-strength and slightly expanding cement-based grout. This setup is illustrated in Figure 1; the technology is convenient and widely adopted [5–7]. The performance of the grouted sleeve is crucial to the viability of the structure. Therefore, many scholars have extensively studied different varieties, inner cavity structure, and new defects of grouted sleeve connections performance.

In order to reduce the cost of the grouted sleeves, find suitable grouted sleeves for a specific project. The following scholars developed new varieties of grouted sleeves and studied the influence of the rebar diameter, anchorage length, and grouting defects on the performance of the grouted sleeves. Seo et al. [8] examined the tensile strength of the grout-filled head-splice-sleeve (HSS) and found that the HSS specimens with no head showed a brittle mortar failure before yielding, whereas the HSS specimens with a suitable head size showed a rebar ductile failure at the end. Lu et al. [9] reported an experimental and analytical study on the mechanical behavior of two kinds of new grouted sleeves processed by seamless steel pipes. The rebar anchorage length was found to be approximately 6–6.4 times the rebar diameter because of the confinement effect. The tensile capacity of the specimens increased with the diameter of the anchorage segment of the rebar as well as the length and slope of the wedge at both ends of the sleeve. Liu et al. [10] investigated the connection performance of restrained deformed grouted sleeve splice. The test showed that the tensile strength of the sleeve splice was equal to the tensile strength of the rebar with an anchorage length eight times the rebar diameter. Yu et al. [11] studied the failure modes, bearing capacity, ductility, and strain distribution of grouted sleeve lapping connectors. The results showed that, with an equal relative lapping length, the yield strength and ultimate load of the specimens increased with an increase in the rebar diameter. The specimens with larger lapping lengths had better initial stiffness and ductility. Chen et al. [12] developed a detectable and repairable half-grouted sleeve (referred to as DDRHGS hereafter). To investigate the tensile performance of the connection using DDRHGS and to validate the reliability of its repair function, five factors were considered comprehensively. The factors were with or without grouting defects, grouting defect ratio, with or without repair material, and rebar diameter. Test results showed that the specimens without defects exhibited a good tensile performance and met the requirements specified in the relevant codes. The grouting defect ratio highly influences the corresponding tensile performance. A higher defect ratio leads to the bond-slip failure mode; the tensile and deformation capacities of such specimens cannot meet the requirements in the relevant codes.

In view of the influence of grouted sleeves inner cavity structure on its performance, the following scholars studied the influence of inner cavity structure and corrosion on the inner wall on mechanical properties of grouted sleeves. Zheng et al. [13] studied the effect of the inner sleeve cavity structure on the bond performance of grouted pipe splice. A direct monotonic pullout test and theoretical analysis showed that increasing the number and height of ribs can improve the tensile capacity of the grouted splice and decrease the displacement of the grouted splice before the rebar yielding. However, a continual increment in the number and height of the rib decreased the effects of varying the inner cavity structure on the bond performance. Du et al. [14] studied the effect of corrosion on the inner wall of the grouting sleeve after a long-term service on its mechanical properties. The test results showed that, at corrosion rates of 0% and 3%, the failure modes of the specimens were rebar fracture. At a corrosion rate of 6% and above, the failure mode was grout pullout, and the ultimate load and ultimate slip decreased with an increase in the corrosion rate. Compared with the noncorroded sleeve, when the corrosion rate reached 12.74%, the ultimate load loss of the specimen was nearly 50%.

Because of the influence of construction technology and environment, grouted sleeves defects became an inevitable problem. The following studies are about the influence of grouting material defects, defects caused by grouting process and different grouting materials on mechanical properties of grouted sleeves. Chen et al. [15] studied the mechanical properties of rebar in half-grouted sleeve connections with water/binder ratio defects. The results illustrated that the failure mode of the specimens with a large diameter was more sensitive to the water/binder ratio, and a considerable decrease in grout strength could occur with an increase in the water/binder ratio. High water/binder ratios led to bond failure and increased the damage depth at the grouting end. Feng et al. [16] studied the bond behavior of deformed rebars in half-grouted sleeve connections with uniform, longitudinal, radial, and inclined grouting defects. The results showed that the specimens underwent the shifting failure mode from the tensile fracture of rebar to the pulling out of rebar with an increase in defect level for all types of grouting defects, especially when the defect level exceeded 30%. Kuang et al. [17] investigated the mechanical properties and deformation of grouted sleeves of different grouting materials through monotonic tension tests under a static force. The authors studied the mechanical performance of the grouted sleeves under minor and major earthquakes through high-stress reversed tension–compression test and large-deformation reversed tension-compression test. The analysis showed that two categories of failure mode could pull out or fracture the rebar; the failure modes were determined by the bond capacity between the rebar and grout as well as the tensile capacity of the rebar. The bond capacity is mainly affected by grout content.

The above studies were mainly focused on connection performance of grouted sleeves in different new forms, inner cavity structure, and various defects. However, in the process of assembling precast concrete components, defects such as rebar offset, rebar bending (see Figure 2), and insufficient fluid grouting material typically occur, because of the production deviation of precast concrete components, improper construction operation, and delay of the grouting job. Therefore, we analyzed the influence of defects above the connection on the performance of half-grouted sleeve connections through uniaxial tension experiments and finite element simulations. Thus, 24 half-grouted sleeve defect specimens were constructed to simulate real construction scenarios.

## 2. Materials and Methods

### 2.1. Materials

High-quality structural steel half-grouted sleeve was used in this study, as shown in Figure 3. The dimensions are shown in Table 1. The mechanical properties of half-grouted sleeve were measured by practical test. Sleeve tensile strength ≥600 MPa, yield strength ≥355 MPa, and elongation ≥15%.

The binder used in the half-grouted sleeve was made of cement-based materials composed of high-strength cement, high-strength fine aggregate, and various polymer additives. The grouting material had several advantages, such as early strength, high strength, micro expansion, high fluidity, and noncorrosive of rebar. Before formal grouting, test blocks and grout fluid were made under the same conditions to determine whether the grouting material inside the casing reached the expected strength, as shown in Figure 4.

The size of the test blocks was 40 mm × 40 mm × 160 mm; each of the three groups contained 3 blocks. Compression test was performed after curing the blocks under standard conditions (20 ± 2°C and 93% relative humidity), and the average compressive strength was adopted.  Table 2 presents the mechanical properties of the grouting material test blocks at different curing ages (1 day, 3 days, and 28 days). The average compressive strength was 40.7 MPa, 70.5 MPa, and 91.4 MPa, respectively. The initial fluidity of grout should not be less than 300 mm; it should not be less than 260 mm within half an hour. The test results met the minimum requirements imposed by JG/T408-2019 [18].

The 14 mm diameter HRB400 grade rebar was adopted. The material properties of the connected rebar, including yield strength and ultimate strength, were tested, as seen in Figure 5. The properties of the rebar material are shown in Table 3.

### 2.2. Specimens Preparation

According to JGJ355-2015 [19], the defect parameters were set to simulate the problems encountered in real project. Eight half-grouted sleeve groups of specimens (seven groups of defect specimens and a control group) were prepared, with three specimens in each group. Details of the specimens are as follows:

1. Control group: we designed the control group according to the code of the half-grouted sleeve. The threaded and grouting ends were the HRB400 rebar with a 14 mm diameter and anchorage length of 120 mm. The grouting material was completely mixed at a 12% hydration rate to avoid bubbles, and grouting within 40 min after being fully mixed. A rubber plug was used to block the inlet and outlet.
2. Rebar offset specimen: engineering construction quality defects usually cause rebar offset joints through a deviation of the embedded rebar of the lower components from the center of the sleeve. The threaded end rebar was inserted into the center of the sleeve, and the grouting end rebar deviated from the center of the sleeve by 5 mm.
3. Rebar bended specimen: the sleeves of the upper precast components cannot be accurately connected with the embedded rebar extending from the lower components in the process of assembling precast concrete components. Workers often make adjustments by hammering causing rebar bended joints. Three groups of rebar bended specimens were prepared, and the bent area deviated from the center of the sleeve by 20 mm, 40 mm, and 60 mm.
4. Insufficient fluidity of grouting material specimen: when workers mix the grouting material and delay the grouting job, because the grouting material is placed for a long time, beyond the best grouting time, the grouting material gradually hardened, the fluidity is reduced, and the strength of the specimens is affected. Three groups of insufficient fluidity of grouting material specimens were prepared; we fully mixed the grout according to specifications and left the mixture for 15 min, 30 min, and 45 min.

Overall, the specimens prepared were of four types: 1 group control, 1 rebar offset group, 3 rebar bended groups, and 3 insufficient fluidity of grout groups (see Figure 6). All the half-grouted sleeves were the same. The grouting material was of the same type and batch, and the rebar was HRB400 with a 14 mm diameter. Details of the specimens are presented in Table 4.

To prepare the uniaxial tensile specimens, a wooden bracket was produced, specimens were fixed on the bracket, the grouting material was mixed, and grouting was performed. All specimens were vertically fixed on the wooden bracket. The independent grouting method was adopted for vertical members, and uniaxial tension experiment was conducted after 28 days of standard maintenance. The procedure is illustrated in Figure 7.

### 2.3. Experimental Device and Loading Pattern

The WAW-1000B electronic hydraulic universal machine (Figure 8) was used in this experiment. The machine has upper and lower clamps; the specimen was fixed vertically by controlling the lower clamps. To observe the failure of the grouting material, the grouting end was kept downward during loading. The entire test and measurement were conducted under displacement control. The loading rate was 5 mm/min, and the experiment was terminated when the specimens were damaged.

### 2.4. Arrangement of the Measuring Point

During the tensile test process, the load and displacement were automatically recorded by the electronic hydraulic universal machine. Five axial strain gauges (*Z*1–*Z*5) and three circumferential strain gauges (*H*1–*H*3) were symmetrically installed along the sleeve. To measure the strain changes of the rebar during the tensile process, the strain gauges (*R*1–*R*10) were installed on the rebar at the connecting end in the anchorage region, both ends of the sleeve, and the bended area. An automatic data acquisition system was used to monitor the strain changes. A YYU200/25 extensometer was used to measure the slip of the specimen, which was bound to the half-grouted sleeve with an adhesive tape, as illustrated in Figure 9.

## 3. Results and Analysis

### 3.1. Failure Modes

Figure 10 illustrates the failure modes of each specimen. All failure modes were rebar fracture failure or along oblique section fracture failure, and the grouting material of the sleeve port was detached.

No apparent change was observed before the specimen yielded in the control group. After the specimen yielded, cracks appeared on the contact surface between the rebar and grouting material at the grouting end, and the cracks fanned out to the inner wall of the sleeve. As the load increased, the rebar fracture failure occurred at the grouting end and the threaded end. The grouting material was conically detached at the sleeve end (see Figure 10(a)).

In the rebar offset group, no obvious changes were found before the specimen yielding. After yielding, cracks appeared first between the rebar and the grouting material on the side close to the inner wall; the cracks then fanned out in all directions. As the load increased, the cracks gradually expanded. The rebar exhibited fracture and oblique fracture failures. The grouting material was detached in different degrees (see Figure 10(b)).

In the rebar bended group, the bended area of the rebar was straightened before yielding. After yielding, the compressive fracture failure and oblique fracture failure occurred, and a part of the specimens broke at the contact surface between the rebar and grouting material. Compared with the first two groups of specimens, the damage degree of the grouting material was smaller (see Figures 10(c)–10(e)).

In the insufficient fluidity of the grouting material group, with an increase in the load after the specimen yielded, the failure mode of the specimens was the rebar fracture failure at the grouting end. The specimens mainly fractured near the sleeve, and the grouting material cracked and flaked off (see Figures 10(f)–10(h)).

### 3.2. Load-Displacement Curves

Figure 11 illustrates the load—displacement curves of each specimen. The load is the tension, and the displacement is the vertical distance between the loading and the reaction beams (see Figure 6). At the initial loading stage, both the rebar and sleeve were observed to be in the elastic deformation stage. As the load increased, the curve of the specimen with clear defects exhibited different trends. The curves consist of the elastic stage, yielding stage, strengthening stage, and tightening stage, which are similar to those of the rebar under uniaxial tension [20–23].

1. The initial loading stage is elastic, and the load and displacement changed linearly.
2. In the yielding stage, the deformation of reinforcement increased gradually, the grouting material of the sleeve port had a clear splitting crack, and the relative slip increased between the rebar and grouting material.
3. In the strengthening stage, the splitting region of the grout at the sleeve port became larger, and the overall deformation of the specimen increased.
4. In the tightening stage, as the displacement increased, the load increased gradually; the rebar was then pulled apart, and the experiment was terminated. The parameters of each specimen are shown in Table 5.

In the control group, the average yield load, average ultimate load, average yield displacement, and average ultimate displacement were 67.66 kN, 93.48 kN, 9.92 mm, and 52.57 mm, respectively. The curves overlapped in three stages of elasticity, yielding, and strengthening, while the stiffness of the specimens was the same. After the grouting material cracked, the development degree of cracks in the axial direction differed, and the bonding strength between the rebar and the grouting material decreased. In the tightening stage, the decline rate of each curve differed with the decrease in the bonding strength (see Figure 11(a)).

In the rebar offset group, the average yield load, average ultimate load, average yield displacement, and average ultimate displacement were 67.59 kN, 92.06 kN, 9.88 mm, and 50.71 mm, respectively. Before the specimen yielding, the curves trend and the stiffness were the same. The curve rose at different rates when it reached its yield point. Afterward, it showed different downward trends after yielding, which was mainly because of the uneven distribution of grout caused by rebar offset. Moreover, the stress difference between the grouting material on both sides of the reinforcement was large when the specimen was under tension (see Figure 11(b)).

In the rebar bended group, the average ultimate loads were 93.44 kN, 91.01 kN, and 82.47 kN, and average ultimate displacements were 71.42 mm, 70.07 mm, and 61.59 mm, respectively. During the loading process, the curve was not apparent at the yielding stage, and it directly entered the strengthening stage after the elastic stage. In addition, the greater the bended degree of the specimen, the smaller the stiffness of the specimen. This relationship existed because the specimen not only bore the axial tension, but also bore the influence of torque and shear force in the tensile process (see Figures 11(c)–11(e)).

In the insufficient fluidity of the grouting material group, the average yield loads were 69.64 kN, 67.70 kN, and 64.97 kN, and the average ultimate loads were 93.20 kN, 91.02 kN, and 90.62 kN, respectively. The average yield displacements were 11.23 mm, 10.60 mm, and 9.74 mm, and average ultimate displacements were 53.30 mm, 51.60 mm, and 48.02 mm, respectively. The variation trend of the curve was roughly the same as that of the control group. Because the fluidity of grouting material was insufficient, the bonding stress between the grouting material, rebar, and sleeve was reduced, and the overall strength of the specimen was lower than that of the control group (see Figures 11(f)–11(h)).

Figure 11(i) illustrates a comparison of load-displacement curves among different specimens. Except for the rebar bended group, the curve variation trend and stiffness are approximately the same. In the early loading process, the bended area is straightened first, and its displacement variation is greater than that of other specimens. Moreover, the greater the degree of the rebar bended, the faster the curves enter the strengthening stage.

All rebar failure modes were rebar fracture failure or along oblique section fracture failure. In the GT14-BM, the specimens were subjected to axial tension during tensile, so the reinforcement showed fracture failure. In other groups of specimens, because of rebar offset and bended, when the specimen is subjected to tensile load, the rebar not only is subjected to axial tensile force, but also is subjected to torque and shear force. These forces can result in undesired stress on the rebar and nonuniform stress distribution in the section of the rebar. As a result, the failure modes were rebar along oblique section fracture failure.

Note: *P*_*y*_ denotes the yield load, *δ*_*y*_ denotes the yield displacement, *f*_*y*_ denotes the yield stress, *P*_*u*_ denotes the ultimate load, *δ*_*u*_ denotes the ultimate displacement, *f*_*u*_ denotes the ultimate stress, $\bar{P_{y}}$ denotes the average yield load, $\bar{\delta_{y}}$ denotes the average yield displacement, $\bar{f_{y}}$ denotes the average yield stress, $\bar{P_{u}}$ denotes the average ultimate load, $\bar{\delta_{u}}$ denotes the average ultimate displacement, and $\bar{f_{u}}$ denotes the average ultimate stress.

### 3.3. Load-Slip Curves

Figure 12 presents the load–slip curves of the specimens. Before the specimen yielding, the slip of the rebar bended specimen increased faster than that of other specimens, and the slip was more than 5 mm. Other specimens were in an elastic state, the curves followed a linear response, and the slips were less than 1 mm. After yielding, different specimens exhibited different trends, and the amount of slip of the rebar bended specimens increased slowly compared with that of other specimens. When the ultimate load was attained, the curves started declining at different rates. The maximum slip of the rebar offset specimen was clearly greater than that of other specimens, and the slip of the rebar bended specimen increased with the bending degree. The flow performance of the grouting material also had a considerable influence on the slip of the specimen. This was mainly because the friction resistance and mechanical bite force between the grouting material, rebar, and sleeve are reduced, and the ability of the specimen to resist deformation was weakened [24–26].

### 3.4. Load-Stress Curves

The typical load–stress curves are shown in Figure 13. The stress is positive for tensile stress and negative for compressive stress. The axial stress of all specimens was tensile stress, while the circumferential stress was mainly compressive stress. Because the crack of grouting material results in volume expansion, the annular contraction of the sleeve restrains its expansion. The combination of the two states determines the stress state on the sleeve. That is, the positive stress indicates that the expansion effect of grout is greater than the constraint effect of the sleeve. On the contrary, the stress is negative [7, 27, 28].

In the control group, the maximum axial tensile stress was approximately 157.15 MPa, and the maximum circumferential compressive stress was approximately 33.35 MPa. Before the specimen yielding, the axial and circumferential stress always followed a linear response. After the specimen yielded, the load continually increased, while the stress gradually decreased, and the curves followed a nonlinear response and rebound. The circumferential stress at *H*3 was changed from compressive stress to tensile stress, mainly because the volume expansion of grouting material after splitting changed the circumferential stress from negative to positive.

In the rebar offset group, the maximum axial tensile stress was approximately 220.73 MPa, and the maximum circumferential compressive stress was approximately 60.67 MPa, which were substantially greater than those of the control group specimens. The main reason for this large difference was that, during the tensile process of the rebar offset specimen, the stress near the cylinder wall was greater than that far from the cylinder wall. Furthermore, the curves followed a linear response before the specimen yielding. The axial tensile stress at Z3 decreased sharply, and the circumferential stress at *H*1 changed from negative to positive when the specimen yielded.

In the rebar bended group, the maximum axial tensile stress was approximately 140.57 MPa, and the maximum circumferential compressive stress was approximately 41.87 MPa, which were less than those of the control group specimens. The axial tensile stress rebound range was wider than that of the control group specimens. The circumferential compressive stress of some specimens increased spirally between positive and negative values with an inflection point. Hence, the bearing capacity increased briefly after the specimen yielded, which was mainly caused by the complex stress state of the specimen during the tensile process.

In the insufficient fluidity of grout group, the maximum axial tensile stress was approximately 134.7 MPa, and the maximum circumferential compressive stress was approximately 34.33 MPa. The curves of some measuring points fluctuated before yielding; after the specimen yielded, it exhibited different rebound trends. At the same time, the specimen bearing capacity decreased.

The stress of all specimens was less than the yield stress of the sleeve, indicating that the sleeve was in an elastic working stage and met the strength requirements. In the uniaxial tensile process, both the axial tensile stress and the circumferential compressive stress increased linearly. Because the rebar entered the stage of plastic deformation, the load–stress curves followed a nonlinear response after the specimen yielded [29].

### 3.5. Stress Distribution Curves

Figure 14 presents the stress distribution curves of the sleeve and rebar at different axial positions under the loading of 20 kN, 40 kN, and 60 kN in specimens GT14-BM-1, GT14-PX-5-3, GT14-WZ-40-3, and GT14-LD-30-1 (they are not all listed because of space limitation). The two stress distribution curves are similar to the inclined roof shape; particularly, the GT14-WZ-40-3 curve fluctuates considerably and has an obvious “inflection point” in the bended area. This observation is mainly because the rigidity and resistance to deformation of rebar reduce after bending. Additionally, it can be observed that the stress of the grouting end rebar in the nonanchorage region was greater than that in the anchorage region, and the stress gradually decreased with an increase in anchorage depth. The maximum sleeve stress was near the threaded end, while the minimum was near the grouting end, which increased with anchorage depth of rebar at the grouting end. It can be concluded that, under the action of high strength load, much of the stress of the half-grouted sleeve connections was borne by the sleeve and grouting material, and the stress of the rebar inside the sleeve was small. Therefore, the connection strength of prefabricated components can be guaranteed in practical engineering.

## 4. Finite Element Analysis

Currently, the detection technology of grouted sleeve in China is not mature. Hence, it is necessary to study the mechanical properties of grouted sleeve in various conditions through finite element analysis. It is also necessary to study the failure mechanism of grouting sleeve through relevant experiments. A finite element software named ABAQUS was used to simulate and analyze the half-grouted sleeve connections, and the reliability of the test and simulation was verified by comparing the load—displacement curves.

### 4.1. Material Constitutive Model

No mature constitutive model exists for the stress-strain relationship of grouting materials. As its properties are similar to those of high-strength concrete, the constitutive relationship of grouting material is typically selected according to high-strength concrete [30]. The concrete plastic damage model selected in this simulation is based on the stress-strain curves of concrete under uniaxial tension and uniaxial compression optimized by GB50010-2010 [31]; the constitutive relationships are shown in Figure 15.

The grouting material compressive strength was 91.4 MPa, the density was 2500 kg/m^3^, the elastic modulus was 38000 MPa, and the Poisson's ratio was 0.2. The density of half-grouted sleeve was 7300 kg/m^3^, the elastic modulus was 2.1 × 10^5^ MPa, and Poisson's ratio was 0.3. The ideal elastic model was adopted; the stress-strain relationship curve is shown in Figure 16. The stress-strain curve of reinforcement is shown in Figure 17. The average yield strength was 420 MPa, the average ultimate strength was 600 MPa, the density was 7850 kg/m^3^, the elastic modulus was 2.0 × 10^5^ MPa, and Poisson's ratio was 0.3.

### 4.2. Finite Element Model

The grouting material, sleeve, and rebar in the model used C3D8R element, all parts of the model as shown in Figure 18. The grouting material, sleeve, and rebar at the grouting end were set in contact; the friction coefficient was 0.2, and the “tie” constraint was set between the rebar at the threaded end with the sleeve.

### 4.3. Finite Element Analysis Results

The test results were compared with the finite element analysis results.  Figure 19 illustrates the load-displacement curve of the rebar offset specimen and rebar bended specimen. As it was difficult to determine the parameters of grouting material beyond the optimal grouting time, the insufficient fluidity of grouting material specimens was not analyzed. The figure illustrates that the finite element analysis results had the same trend as the test results. Because the constraint mode set between sleeve, grouting material, and rebar in simulation could not ensure the complete consistency with the test. Furthermore, owing to the cracking of grouting material in different degrees, a relative slip was observed between the rebar and grouting material. The yield and ultimate loads of the specimen after finite element analysis were slightly larger than those of the test [32, 33]. The numerical simulation result of the yield load of the rebar offset specimen was 68.64 kN, the ultimate load was 85.59 kN, and the numerical simulation results of the ultimate load of the rebar bended specimens were 90.18 kN, 88.50 kN, and 80.34 kN, respectively. Compared with the test results with the same parameters, the errors were all less than 8%, indicating that the simulation results were consistent with the test results. Thus, the correctness of the numerical model and the rationality of the key parameters were verified.

Figure 20 presents the finite element stimulation stress distribution diagram of joint, grouting material, and sleeve. The maximum stresses of the sleeve were 445.62 MPa. The maximum stresses of rebar were 586.10 MPa. The maximum stress of the rebar bended specimen was in the bended area, which is consistent with the test results.

The yield and ultimate loads of the numerical simulation were compared with those of the test as shown in Table 6. Compared with the experimental results, the deviations of yield and ultimate loads in the numerical simulation were within 8%. This was because the constitutive model of the grout material in simulation could not perfectly replace the constitutive relation of the experiment.

## 5. Conclusion

In this study, we examined the mechanical properties of eight groups of half-grouted sleeve joints in three kinds of construction defects. The main findings from the experimental observations are as follows:

1. The failure mode of all half-grouted sleeve specimens was rebar fracture failure. Except the rebar bended specimens, the load-displacement curves consisted of elastic, yielding, strengthening, and tightening stages, which were similar to those of rebar under uniaxial tension.
2. In the tensile process, there was no obvious yield stage in the load-displacement curves of the rebar bended specimens. The curve directly entered the strengthening stage from the elastic stage. As the bending section increased, the rigidity and resistance to deformation of rebar bended specimens decreased.
3. The axial stress of the sleeve exhibited a linear response before yielding, and it rebounded after yielding because of the plastic deformation of the rebar at the grouting end. Owing to the expansion of the grouting material and the circumferential contraction of the sleeve, the circumferential stress may be tensile stress or compressive stress.
4. The axial stress of the sleeve increased with the rebar anchorage depth at the grouting end. The rebar stress in the sleeve cavity decreased with increasing anchoring depth, and the stress in the nonanchorage region was greater than that in the anchorage region.
5. The finite element analysis results showed that the ultimate load and stress distribution of the specimen coincided with those of the experimental results, and the deviations were within 5%.

## Figures and Tables

**Figure 1:** Prefabricated concrete component connection using half-grouted sleeves.

**Figure 2:** Rebar bending.

**Figure 3:** Axial profile of half-grouted sleeve.

**Figure 4:** Grout properties test.

**Figure 5:** Rebar properties test.

**Figure 6:** Details of the specimens (unit: mm). (a) GT14-BM, (b) GT14-PX-5, (c) GT14-WZ-20, (d) GT14-WZ-40, (e) GT14-WZ-60, and (f) GT14-LD.

**Figure 7:** Experimental procedure.

**Figure 8:** Experimental device.

**Figure 9:** The arrangement of the measuring point. (a) Arrangement of strain measuring points (unit: mm). (b) Automatic data acquisition system. (c) Extensometer arrangement.

**Figure 10:** Failure modes. (a) GT14-BM, (b) GT14-PX-5, (c) GT14-WZ-20, (d) GT14-WZ-40, (e) GT14-WZ-60, (f) GT14-LD-15, (g) GT14-LD-30, and (h) GT14-LD-45.

**Figure 11:** Load-displacement curves. (a) GT14-BM, (b) GT14-PX-5, (c) GT14-WZ-20, (d) GT14-WZ-40, (e) GT14-WZ-60, (f) GT14-LD-15, (g) GT14-LD-30, (h) GT14-LD-45, and (i) curves contrast.

**Figure 12:** Load-slip curves. (a) GT14-BM, (b) GT14-PX-5, (c) GT14-WZ-20, (d) GT14-WZ-40, (e) GT14-WZ-60, (f) GT14-LD-15, (g) GT14-LD-30, (h) GT14-LD-45, and (i) curves contrast.

**Figure 13:** Load-stress curves. (a) GT14-BM-1, (b) GT14-PX-5-3, (c) GT14-WZ-20-2, (d) GT14-WZ-40-3, (e) GT14-WZ-60-3, (f) GT14-LD-15-2, (g) GT14-LD-30-1, and (h) GT14-LD-45-3.

**Figure 14:** Stress distribution curves. (a) GT14-BM-1, (b) GT14-PX-5-3, (c) GT14-WZ-40-3, and (d) GT14-LD-30-1.

**Figure 15:** Stress-strain curve of grout. (a) Uniaxial compression of concrete. (b) Uniaxial tension of concrete.

**Figure 16:** Sleeve stress-strain curve.

**Figure 17:** Rebar stress-strain curve.

**Figure 18:** The finite element model. (a) GT14-PX-5, (b) GT14-WZ-20, (c) GT14-WZ-40, and (d) GT14-WZ-60.

**Figure 19:** Load-displacement curves. (a) GT14-PX-5, (b) GT14-WZ-20, (c) GT14-WZ-40, and (d) GT14-WZ-60.

**Figure 20:** The finite element stimulation stress distribution diagram. (a) GT14-PX-5, (b) GT14-WZ-20, (c) GT14-WZ-40, and (d) GT14-WZ-60.

**Table 1:** Half-grouted sleeve parameters.

Serial number	*L/*mm	*L*_1_/mm	*L*_2_/mm	*D*_1_/mm	*D*_2_/mm	*d*_1_/mm	*d*_2_/mm	*d*_3_/mm	*t*/mm
GT14/14	155	25	130	34	30	16	14	14	2

**Table 2:** Mechanical properties of grouting material at different curing ages.

Curing age (d)	Specimens (d)	Compressive strength/MPa	Average/MPa	Standard/MPa
1	1–1	40.1	40.7	≥35
	1–2	40.6		
	1–3	41.3		

3	3–1	70.3	70.5	≥60
	3–2	71.5		
	3–3	69.8		

28	28–1	91.2	91.4	≥85
	28–2	90.8		
	28–3	92.3		

**Table 3:** HRB400 rebar material properties.

Specimens	1	2	3	Average	Standard
Rebar diameter/mm	14	14	14	14	/
Yield strength/MPa	418	423	409	417	400
Tensile strength/MPa	593	586	595	591	540

**Table 4:** Details of the specimens.

Types	Specimen's number	Defect parameters	Number
Control group	GT14-BM-1/2/3	/	3

Rebar offset	GT14-PX-5-1/2/3	Grouting end rebar deviated from the center of the sleeve 5 mm	3

Rebar bended	GT14-WZ-20-1/2/3	Grouting end rebar bended 20 mm	3
	GT14-WZ-40-1/2/3	Grouting end rebar bended 40 mm	3
	GT14-WZ-60-1/2/3	Grouting end rebar bended 60 mm	3

Insufficient fluidity of grouting material	GT14-LD-15-1/2/3	Grouting material stood for 15 min	3
	GT14-LD-30-1/2/3	Grouting material stood for 30 min	3
	GT14-LD-45-1/2/3	Grouting material stood for 45 min	3

**Table 5:** Experimental feature point.

Specimen's number	*P*_*y*_/kN	*δ*_*y*_/mm	*f*_*y*_/MPa	*P*_*u*_/kN	*δ*_*u*_/mm	*f*_*u*_/MPa	$\bar{P_{y}}$ /kN	$\bar{\delta_{y}}$ /mm	$\bar{f_{y}}$ /MPa	$\bar{P_{u}}$ /kN	$\bar{\delta_{u}}$ /mm	$\bar{f_{u}}$ /MPa
GT14-BM-1	68.13	9.82	442.58	93.47	53.68	607.19	67.66	9.55	439.55	93.48	52.57	607.28
GT14-BM-2	66.92	8.93	434.72	93.49	50.86	607.32						
GT14-BM-3	67.94	9.89	441.35	93.49	56.18	607.32						

GT14-PX-5-1	69.27	10.30	449.98	93.48	48.48	607.26	66.59	9.88	432.57	92.06	50.71	598.01
GT14-PX-5-2	66.42	10.76	431.47	90.97	49.43	590.95						
GT14-PX-5-3	64.08	8.58	416.27	91.72	54.21	595.82						

GT14-WZ-20-1	/	/	/	93.65	75.29	608.36	/	/	/	93.44	71.42	606.57
GT14-WZ-20-2	/	/	/	92.84	69.51	601.80						
GT14-WZ-20-3	/	/	/	93.84	69.46	609.60						

GT14-WZ-40-1	/	/	/	91.50	72.08	594.39	/	/	/	91.01	70.07	591.23
GT14-WZ-40-2	/	/	/	90.61	71.42	588.61						
GT14-WZ-40-3	/	/	/	90.93	72.72	590.69						

GT14-WZ-60-1	/	/	/	79.97	62.60	519.49	/	/	/	82.47	61.58	533.57
GT14-WZ-60-2	/	/	/	84.73	55.38	550.42						
GT14-WZ-60-3	/	/	/	82.71	66.78	530.80						

GT14-LD-15-1	69.83	12.95	453.62	93.73	57.58	608.88	69.94	11.13	454.34	93.20	53.3	605.45
GT14-LD-15-2	69.28	9.32	450.05	93.90	50.62	609.98						
GT14-LD-15-3	70.71	11.12	459.34	91.96	51.70	597.38						

GT14-LD-30-1	66.78	11.40	433.81	91.22	54.04	592.58	67.70	10.60	439.77	91.02	51.60	591.3
GT14-LD-30-2	66.85	10.07	434.27	91.35	51.19	593.42						
GT14-LD-30-3	69.46	10.33	451.22	90.50	49.58	587.90						

GT14-LD-45-1	63.71	9.68	413.87	89.68	50.21	582.57	64.97	9.74	422.07	90.62	48.02	588.67
GT14-LD-45-2	67.13	10.02	436.08	90.36	49.03	586.98						
GT14-LD-45-3	64.08	9.52	416.27	91.82	44.81	596.47						

**Table 6:** Test and FEA result contrast.

	Specimen	GT14-BM	GT14-PX-5	GT14-WZ-20	GT14-WZ-40	GT14-WZ-60
Yield load/kN	Experiment	67.66	66.59	/	/	/
	FEA	70.52	68.64	/	/	/
	Deviation	4.23%	3.07%	/	/	/

Ultimate load/kN	Experiment	93.48	92.06	93.44	91.01	82.47
	FEA	97.45	85.59	95.83	95.54	85.86
	Deviation	4.25%	7.03%	3.49%	2.76%	3.02%

## Data Availability

All data generated or used during the study are available within the article.
